The article "The Relationship between Sleep Quality and Hemodialysis and Nursing Intervention in Uremia Patients Based on Intelligent Data" was retracted in 2023. Reasons: suspected computer-generated content; unreliable results or conclusions; lack of ethics approval or compliance; missing or withdrawn patient consent.

# The Relationship between Sleep Quality and Hemodialysis and Nursing Intervention in Uremia Patients Based on Intelligent Data

**DOI:** 10.1155/2022/3211144

**Published:** 2022-07-25

**Authors:** Aixia Lin, Fujuan Zhang, Huifang Zhang

**Affiliations:** ^1^Hemodialysis Room, Yantai Mountain Hospital, Yantai, 264001 Shandong, China; ^2^Delivery Room of Shandong Provincial Hospital Affiliated to Shandong First Medical University, Jinan, 250000 Shandong, China

## Abstract

Uremia is a manifestation of end-stage renal failure and is a clinical syndrome shared by various advanced renal diseases. In recent years, the prevalence of uremia has been increasing. Maintenance hemodialysis therapy is used as the treatment of choice for uremia and is widely used. For uremia, the day-to-day treatment has a serious impact on the patient's symptoms, causing a lot of unnecessary burdens to life. While imposing a severe symptom burden on patients, excessive sleep deprivation repair time can cause various risk injuries and further increase the probability of patient mortality. The resulting sleep deprivation can lead to the functional damage of multiple organs and systems such as the cardiovascular system and the immune system. Therefore, improving sleep quality can increase the survival rate of patients to a certain extent. There is less domestic attention to its related research, and there are not many discussions on the pathogenesis. Based on this, this paper proposes to explore the effect of hemodialysis on the sleep quality of patients with uremia under the support of intelligent data. In this study, it was found that MHD patients had various sleep quality problems, and the incidence of sleep disturbance was 61.78%. The experimental results in this paper show that the incidence of sleep disturbance in diabetic nephropathy is 89.7%. This may be combined with a series of complications in patients with diabetes, which in turn affects the quality of sleep in patients. It may increase patient mortality and affect patient quality of life and survival. Therefore, we should pay close attention to the prevention of various complications in diabetic dialysis patients, which will help to improve sleep quality.

## 1. Introduction

Chronic kidney disease (CKD) is an increasing public health problem, because of its increasing morbidity and mortality and significantly increasing the risk of cardiovascular disease, resulting in huge medical costs. With regard to maintenance hemodialysis (MHD), it is inevitable that we must face a big problem. As for maintenance hemodialysis, it is inevitable that we must face a big problem. The quality of life and survival rate of this special group of MHD patients should be paid more attention. As the most common complication of MHD patients, sleep disturbance should be paid more and more attention. There are many factors that affect sleep quality in MHD patients. At present, there are not many domestic researches in this area. Hospital X, as the most influential tertiary first-class general hospital in the region, has relatively concentrated MHD patients, and the cases are also representative to a certain extent. Therefore, this study adopts a field survey. The results of statistical analysis can guide us to prevent or eliminate risk factors associated with sleep disorders. Actions that can be taken include the following: the investment in social security can be strengthened, the WeChat group and QQ group of patients can be established, and a chronic kidney disease management group can be established. It can strengthen the communication between doctors and patients, between patients, and between patients and their families. All kinds of problems need to be dealt with immediately, and psychological counseling should be carried out in a targeted manner. It can regularly carry out patient health education and dietary guidance and conduct popular science education for patients and their families. Patients can be guided to the correct intake of sodium, calcium, phosphorus, water, etc. It is necessary to emphasize the individualized dialysis program and choose an economical combination of dialysis.

Chronic kidney disease has become a global public health problem, and the number of people receiving renal replacement therapy is increasing rapidly every year. With the improvement of the social medical security system, the promotion of ESRD special diseases and single-disease payment, and the general lack of transplanted kidney sources, it is foreseeable that the number of MHD patients will increase year by year. And its incidence will increase in the next two decades. The prevalence of sleep disturbances is generally higher in MHD patients. The decline of sleep quality directly leads to the decline of the quality of life of MHD patients. Its main manifestations are easy to wake up, poor sleep quality, insomnia, long-term dependence on hypnotic drugs, and sleep apnea. The problem of sleep quality in MHD patients has become an important factor that threatens patients' lives and long-term survival. As for improving the patient's sleep quality, it will help to improve the patient's life and quality of life. Therefore, the investigation and intervention of patients' sleep quality and its influencing factors should be paid more and more attention.

This study investigated the status of sleep disturbances (including overall sleep quality and classified sleep disturbances) in maintenance hemodialysis patients. It found a number of modifiable factors such as age, dialysis months, interdialysis weight gain, and dialysis methods. This can guide clinical caregivers to personalize sleep hygiene interventions for patients, thereby improving patients' sleep problems. This study provides clues and basis for further implementation of analytical research and interventional research on sleep disorders in maintenance hemodialysis patients. It also discussed its effect on sleep disturbance in maintenance hemodialysis patients and reached meaningful conclusions, which can provide reference for follow-up research.

## 2. Related Work

Maintenance hemodialysis is an important way to prolong the life of patients with uremia. In recent years, kidney disease has frequently occurred, which is one of the important reasons for the increase in mortality of patients. Scholars from all over the world have made corresponding explorations on the pathology of maintenance hemodialysis patients. Zhao's paper on the relationship to sclerostin in relation to circulatory incidents as well as cardiac mortality of people on dialysis cites several studies for comparison. Consistency of testing methods should be standardized [1]. Samy evaluated association with serum magnesium in hemodialysis patients with changes in atherosclerosis. It was concluded that serum magnesium can be regarded as a changeable weight risk element for arterial coagulation in patients on hemodialysis [2]. Hishii investigated an association in chronic hemodialysis patients between sitting behavior as well as health-related quality of life (HRQOL). The regression results further showed that reducing sedentary behavior may be beneficial in improving HRQOL in chronic hemodialysis patients [3]. Aghsaiefard investigated associations between both anemia and parathyroid hormone among chronic hemodialysis patients and dialysis adequacy. The results of his investigation showed that decreased hemoglobin values lead to decreased erythropoietin resistance. Correlates of serum levels of iron, a gross total binding capacity (TIBC) as well as erythropoietin tolerance with hematocrit levels [4]. Lu studied the relationship between changes in blood pressure during dialysis and all-cause mortality as well as cardiovascular mortality. Exploration showed that MHD patients with significantly elevated blood pressure after hemodialysis had a higher risk of death [5]. Gulin further compared the prevalence of inpatient and out-of-hospital hemodialysis (HD) clients with regard to the prevalence of ambulatory hypertension as well as changes in their blood pressure (BP) during HD. The results showed differences in BP changes and antihypertensive therapy between inpatient and out-of-hospital dialysis patients, reflecting the different practices of kidney physicians in those centers [6]. Seefried assessed whole body vibration exercise (WBV). The safety and efficacy of improving physical performance and inflammatory parameters in maintenance hemodialysis (MHD) patients. Conclusion: the results of the study demonstrate the efficacy and safety of WBV in hemodialysis patients [7]. Many scholars have carried out corresponding research on uremic hemodialysis patients. They mostly use actual patient cases as research objects, and the sample collection points are mostly in one place. Therefore, patients who are the same and not affected by other diseases are not easy to aggregate, and most patients have other diseases. This makes the exploration process have certain discrepancies and easily affects the research results.

## 3. The Relationship between Hemodialysis and Sleep Disorders in Uremia Patients Based on Intelligent Data

### 3.1. Epidemiology of End-Stage Renal Disease

Uremia is a clinical stage in which various primary or secondary renal diseases progress to irreversible loss of renal function. Severe uremic symptoms can lead to a decline in quality of life and the end of the life course [8]. From a global perspective, the prevalence of end-stage renal disease is still increasing year by year, but the incidence has entered a plateau since 2000 and has declined in the past two years. At present, there is still a lack of real-time, effective, and comprehensive uremia-related statistical data in China. Taiwan and Hong Kong participated in the data statistics of the US Kidney Disease Data System.

As of December 31, 2011, the prevalence of uremia in Taiwan ranked first. From 2003 to 2010, among the etiological composition of 7474 new hemodialysis patients in China, the proportion of chronic glomerulonephritis decreased, while the proportion of diabetes gradually increased [9]. With the aging of the population and the prolongation of the survival period of primary diseases such as diabetes, hypertension, and obesity, the prevalence of uremia is increasing year by year. Although the main cause is currently glomerular disease, it is expected that in the next few years, diabetes and hypertension will gradually become the main causes. Therefore, we are faced with the dual challenges of traditional diseases and diseases related to poor lifestyle [10].

Application of hemodialysis: at present, the feasible treatment method for end-stage renal disease is renal replacement therapy [11]. This identified effective alternatives including hemodialysis, peritoneal dialysis, and kidney transplantation. As the main form of renal replacement therapy, hemodialysis has been rapidly developed and popularized in recent years [12]. The principle of hemodialysis is shown in Figure 1, which can effectively prolong the survival of uremia patients.  Figure 2 shows the basic flow for hemodialysis patients. It can be found through the process that all aspects of hemodialysis require strict evaluation and review. However, hemodialysis treatment itself has many problems [13]. For example, hypotension, vomiting, and muscle disease may occur during dialysis, and the long interval between two dialysis may increase the risk of death in dialysis patients. And with the extension of dialysis years, complications are also increasing. Sleep disturbance is one of the issues that has been widely discussed in recent years [14]. According to a research report, sleep disturbance is one of the six most troublesome symptoms of hemodialysis patients, and the prevalence rate is as high as 86%. This seriously affects the quality of life of patients and increases the risk of death in dialysis patients and affects disease prognosis [15].

### 3.2. The Concept of Sleep Disorders

(1) Related concepts and classifications of sleep disorders: sleep disturbances are sleep-related abnormalities in humans or other animals. To be precise, sleep disorder refers to a state of dissatisfaction with the quality and quantity of sleep for a period of time [16].  Figure 3 shows the specific manifestations of sleep disorders

What needs to be differentiated from sleep disorders is the concept of sleep deprivation [17]. Sleep deprivation refers to a state in which a person cannot get enough sleep due to environmental or personal reasons. Often sleep deprivation can have adverse effects on various systems and organs throughout the body, such as this will increase the risk of cardiovascular disease and reduce immune function. This has many adverse effects on the prognosis of hemodialysis patients [18]. As mentioned earlier, sleep disturbance is a very broad concept. It can refer to a variety of other sleep problems.

### 3.3. BP Learning Algorithm

The BP algorithm is composed of a learning process consisting of two processes: forward propagation of the signal and backward propagation of the error. The BP neural network has rekindled the enthusiasm for deep learning. It solves the calculation problem of weight values in hidden layer transfer in DNN. It is a multilayer feedforward neural network trained according to the error backpropagation algorithm.

Usually, the expected output value in the network is not equal to the actual output result, and there is a certain error between them [19]. It denotes this error as *C*, and its basic definition is as follows:

(1) $$\begin{array}{c} C=\frac{1}{2}{\left(b-0\right)}^{2}=\frac{1}{2}\overset{i}{\underset{e=1}{\sum }}{\left(be-0e\right)}^{2}. \end{array}$$

To adjust the weights of the BP neural network, it should follow the principle of reducing the error. Therefore, the number of adjustment weights ought to be directly related with respect to the negative grade of uncertainty [20], which can be expressed as

(2) $$\begin{array}{c} \Delta Mie=-\beta \frac{\alpha C}{\alpha \text{net}e}\frac{\alpha \text{net}e}{\alpha Mie},\;i=1,2,\cdots ,n,\\ \Delta Nih=-\beta \frac{\alpha C}{\alpha \text{net}i}\frac{\alpha \text{net}i}{\alpha Mih},\;h=1,2,\cdots ,m. \end{array}$$

Meanwhile, the difference in error function can be

(3) $$\begin{array}{c} C=\frac{1}{2}\overset{i}{\underset{e=1}{\sum }}{\left[be-j\left(\overset{r}{\underset{h=1}{\sum }}Miefh\right)\right]}^{2}. \end{array}$$

The weight adjustment from the hidden layer to the output layer in the network can be expressed as

(4) $$\begin{array}{c} \Delta Mim=\beta \left(be-0e\right)j^{\prime }\left(\text{net}e\right)Bf. \end{array}$$

The weight adjustment formula from the input layer to the hidden layer in the network can be expressed as

(5) $$\begin{array}{c} \Delta Nih=\beta \overset{r}{\underset{h=1}{\sum }}\left[\left(be-0e\right)j\left(\text{net}e\right)Mie\right]j^{\prime }\left(\text{net}i\right)Ar. \end{array}$$

The sigmoid function is used for the output of hidden layer neurons, and the value range is (0, 1). It can map a real number to the interval (0, 1) and can be used for binary classification. It also uses the sigmoid function, that is,

(6) $$\begin{array}{c} j\left(A\right)=\frac{1}{1+\exp\left(-A\right)},\\ j^{\prime }\left(A\right)=j\left(A\right)\left[1-j\left(A\right)\right]. \end{array}$$

Then,

(7) $$\begin{array}{c} \Delta Mie=\beta \left(be-0e\right)0e\left(1-0e\right)Bi,\\ \Delta Nih=\beta \overset{r}{\underset{h=1}{\sum }}\left[\left(be-0e\right)0e\left(1-0e\right)Mie\right]Bi\left(1-Bi\right)Ai. \end{array}$$

All training samples are referred to as a training epoch for each input. When training a neural network using the backpropagation algorithm, there are two options available [21]. One is to modify the weights each time a sample is input, which is called one-shot training [22]. This method only adjusts for the error produced by the current sample. It inevitably leads to an increase in the number of training sessions, and the convergence rate is too slow. The other is that of a batch process approach, where the total average mistake is calculated at the end of a single instance of training [23].

(8) $$\begin{array}{c} Cxn=\frac{1}{2V}\overset{v}{\underset{i=1}{\sum }}\underset{e}{\sum }c_{e}^{2}\left(i\right), \end{array}$$

where *C*_*e*_^2^(*i*) represents the error under *i* input samples of the *e*-th output unit and *V* represents the total number of all training sample sets.

The steps of the backpropagation algorithm can be summarized as follows:

(1) Initialization: the initial error *C* is assumed to be 0, and the learning rate *β* is expressed as a decimal between 0 and 1 [24]
(2) The input samples are computed in a front-to-back order to obtain the results of the hidden layer and the output layer
  (9) $$\begin{array}{c} \text{net}i=\overset{j}{\underset{i=1}{\sum }}NijAi,\;i=1,2,\cdots ,n,\\ Bi=j\left(\text{net}i\right),\;i=1,2,\cdots ,n,\\ {\text{net}}_{e}=\overset{n}{\underset{f=1}{\sum }}MieBi,\;e=1,2,..,m,\\ 0e=j\left(\text{net}e\right),\;e=1,2,\cdots ,m. \end{array}$$
(3) If one cycle of training ends, that is, all *R* samples have participated in one round of training, go to step 2
(4) It calculates the error signal of each layer according to the total error
  (10) $$\begin{array}{c} \frac{\alpha \text{C}}{\alpha \text{nete}}=-\frac{1}{V}\overset{v}{\underset{i=1}{\sum }}\left[\left(b_{e}^{1}-0_{e}^{1}\right)j^{\prime }\left({\text{net}}_{e}^{1}\right)\right],\\ \frac{\alpha C}{\alpha \text{net}i}=-\frac{1}{V}\overset{v}{\underset{i=1}{\sum }}\left\{\overset{m}{\underset{e=1}{\sum }}\left[\left(b_{e}^{1}-0_{e}^{1}\right)j^{\prime }\left({\text{net}}_{e}^{1}\right)Mie\right]j^{\prime }\left({\text{net}}_{i}^{1}\right)\right\}. \end{array}$$
(5) It calculates the weight adjustment of each layer
  (11) $$\begin{array}{c} \Delta Mie=\frac{\beta }{V}\overset{v}{\underset{i=1}{\sum }}\left[\left(b_{e}^{1}-0_{e}^{1}\right)j^{\prime }\left({\text{net}}_{e}^{1}\right)B_{i}^{1}\right],\\ \Delta Nih=-\frac{\beta }{V}\overset{v}{\underset{i=1}{\sum }}\left\{\overset{m}{\underset{e=1}{\sum }}\left[\left(b_{e}^{1}-0_{e}^{1}\right)j^{\prime }\left({\text{net}}_{e}^{1}\right)Mie\right]j^{\prime }\left({\text{net}}_{i}^{1}\right)A_{i}^{1}\right\}. \end{array}$$
(6) It modifies the network weights
(7) It checks whether the network accuracy meets the predetermined requirements, and if so, the training ends. If not, it will perform a new one-cycle training

## 4. Hemodialysis and Sleep Quality of Uremia Patients Based on Intelligent Data

### 4.1. Methods

In this paper, the sample collection of uremic hemodialysis patients is concentrated in the departments of X hospital. A total of 157 suitable patients were included in the hospital. The basic age, gender, and disease subdivision collection and classification are shown in Figure 4.

As seen in Figure 4, uremic hemodialysis patients were concentrated between 30 and 60 years of age and were mostly with chronic nephritis and diabetic nephropathy, with the least polycystic kidney and obstructive nephropathy.

### 4.2. Details of Research Methods

This article reviewed the recent medical records of 157 MHD patients in X hospital. It investigates the general condition of MHD patients in the past 1 month, and age, gender, dialysis month, dialysis frequency, dialysis method, dialysis time points, serum albumin levels, cholesterol, triglycerides, hemoglobin, calcium-phosphorus product, serum creatinine level, BNP level, diabetic nephropathy, whether hepatitis B carrier, whether refractory hypertension, and so on [25]. It uses the Pittsburgh sleep quality index (PSQI) scale. The scale is suitable for the evaluation of sleep quality in patients with sleep disorders and psychiatric disorders, as well as for the assessment of sleep quality in the general population. It assessed the sleep quality of 157 MHD patients by means of an onsite questionnaire survey (all in the form of one question and one answer) [26]. The Pittsburgh sleep quality index scale was used to assess the sleep quality of the subjects in the last month. And those with a PSQI total score greater than 5 were recorded as sleep disorders.

In this study, 225 ERSD patients requiring hemodialysis were treated in X hospital from January to September. Among them, 157 MHD patients met the criteria, accounting for 69.78% of the dialysis patients, with an average PSQI value of 5.7 ± 3.3 points. Among them, 97 patients had PSQI index greater than 5 points, accounting for 61.78% of MHD patients. This further confirms that sleep disturbance is a common complication in maintenance hemodialysis patients. It may have a great impact on the survival and quality of life of patients.

### 4.3. Factors Affecting Sleep Quality of Uremia Patients Based on Intelligent Data

In this paper, the basic information of suitable patients in X hospital was collected, and the sleep quality was scored by gender. The statistical results are shown in Table 1.

The prevalence of sleep disorders tends to increase with age. Therefore, this study was divided into 5 groups by age using a span of 15 years. That is, below 30 years old (A), 30-45 years old (B), 45-60 years old (C), 60-75 years old (D), and above 75 years old (E). The prevalence of sleep disorders was 42.9% in group A with 14 cases and 6 cases with PSQI > 5. 45 cases in group B with 20 cases with PSQI > 5, the prevalence was 44.4%. 48 cases in group C with 34 cases with PSQI > 5, the prevalence was 70.8%. 34 cases in group D with 25 cases with PSQI > 5, the prevalence was 73.5%. 17 cases in group E with 12 cases with PSQI > 5, the prevalence was 70.5%. The differences between group A and groups C and D (*P* < 0.05) and between group B and groups C and D (*P* < 0.01) were statistically significant.

As shown in Table 2 and Figure 5, the age of uremic patients affects the quality of sleep. According to the literature, whether the prevalence of sleep disorders in ESRD patients differs by gender varies between national and international studies. In the data in this paper, the prevalence was essentially the same for both genders. This may be related to different regions and ethnic differences, different proportions of social and family responsibilities assumed by men and women, and different personal preferences (e.g., smoking and alcohol consumption).

As shown in Table 2 and Figure 5, the age of uremic patients affects sleep quality. From the literature research, whether there is a difference in the incidence of sleep disorders in ESRD patients of different genders, there are differences in the results of domestic and foreign studies. In the data of this group, there were 104 males and 54 females, with a sex ratio of 1 : 1.93. The average age of men is 2 years older than that of women, but the prevalence of men and women is basically the same. There was no significant difference in the prevalence of sleep disorders between male patients and female patients, which was similar to the results of many domestic studies. This may be related to factors such as different regions, ethnic differences, different proportions of social and family responsibilities undertaken by men and women, and different personal preferences (such as smoking and drinking).

In this study, we analyzed different age groups and found that the sleep quality of dialysis patients between the ages of 45 and 75 was significantly lower than that of other age groups. There was a statistically significant difference between the incidence of sleep disturbances in this age group and other age groups. This may be related to the fact that dialysis patients in the 45-75 age group are the main household labor force in this region. They are affected by major family work, heavy family economic burden, anxiety, depression, and other psychological factors, so the quality of sleep is significantly reduced. Compared with other age groups, the difference was not statistically significant in patients older than 75 years. This may be related to the fact that most of the patients in this age group are not the main labor members of the family. And the survey found that many of these patients are retirees or families with successful careers, with low economic burden, high awareness of children, and low psychological burden. Therefore, improving social security services, reducing the economic burden of MHD patients, strengthening psychological communication, and improving the concern of family members should have a greater effect on improving the sleep quality of patients.

## 5. The Influence of Various Factors on Sleep Quality

### 5.1. The Effect of Dialysis Frequency on Sleep Quality

There were 3 dialysis frequencies in 157 MHD patients, namely, 2 times/week (group A), 5 times/2 weeks (group B), and 3 times/week (group C). Among them, there were 52 cases in group A, 35 cases with PSQI > 5 points, the prevalence rate of sleep disorder was 67.3%; 32 cases in group B, 16 cases with PSQI > 5 points, the prevalence rate was 48.5%, while 75 cases in group C had PSQI > 5 points in 45 cases, the prevalence rate was 60%. Through the comparison among the groups, it was found that there was no significant difference in the prevalence of sleep disorders among the groups (*P* > 0.05). The statistical results and schematic diagrams of *X*^2^ and *P* value changes are shown in Tables 3 and 4 and Figure 6.

The data in Figure 6 has been modified by calculation, and the style of Figure 6 has been modified.

157 patients with MHD were divided into 3 groups. There were 37 cases in group A with a mean dialysis age of 7.4 ± 2.8 months, 18 cases with PSQI > 5 score, and a prevalence of 44.4% for sleep disorders. 47 cases in group B with a mean dialysis age of 24.3 ± 6.8 months, 36 cases with PSQI > 5 score, and a prevalence of 75%. 74 cases in group C with a mean age of 52.2 ± 13.8 months, 45 cases with PSQI > 5 score, and a prevalence of 60%. The prevalence rate was 60%. A comparison between groups revealed a statistically significant difference between group A and group B (*P* < 0.05).

The data in this group showed that the incidence of sleep disturbance was significantly increased in MHD patients with dialysis months between 12 and 36 months. Compared with other dialysis months, the difference was statistically significant. However, after multivariate analysis, it was found that it was not an independent risk factor. Compared with patients in the 12- to 36-month age group and dialysis patients with dialysis time less than 12 months old, patients in this stage have no significant improvement in disease awareness. Their acceptance of the disease remains low. At the same time, due to the increase of their dialysis months, the economic burden gradually increased, the residual renal function decreased, and the anxiety and depression were not improved significantly, so the incidence of sleep disorders was high.

Compared with patients aged 12-36 months and patients with dialysis months older than 36 months, although their economic burden is not as good as the latter, their awareness and psychological acceptance of the disease are not as good as the latter, so the incidence of sleep disorders is also higher. Combining the above factors, we can strengthen the interaction with doctors and patients, between patients, and between patients and their families for each dialysis age group. It is necessary to strengthen disease popularization, clear the psychology, and reduce the psychological burden of patients. It also called on the society to strengthen the care for MHD patients.

During maintenance hemodialysis, the frequency of dialysis in MHD patients is closely related to changes in the patient's economic status and weight gain. It needs to be formulated by the doctor according to the patient's condition and is relatively individualized. The present study found that there was no statistically significant difference in the incidence of sleep disturbance between different dialysis frequencies. This may be related to the fact that all patients in this study were on regular maintenance dialysis. The choice of dialysis frequency may be mainly determined by the patient's weight, the amount of weight gain between dialysis, and the level of creatinine before dialysis. And with the increase of dialysis frequency, the nutritional loss is more obvious, which has a more significant impact on the patient's constitution. Therefore, it is not that the higher the frequency of dialysis, the better the quality of dialysis, and the reasonable frequency of dialysis should fully reflect individual differences and should be adjusted at any time according to the patient's condition.

### 5.2. The Effect of Dialysis on Sleep Quality

Several modalities of dialysis exist in patients with MHD in Hospital X. These are hemodialysis (HD), hemodiafiltration (DHF), and hemoperfusion (HP). According to the dialysis method chosen by the patients, they were divided into 4 groups. These are group A (HD), group B (DHF), group C (HD+HDF), and group D (HD+HP). Among them, there were 86 cases in group A, 65 cases with PSQI > 5 points, and the prevalence of sleep disorder was 75.3%. There were 10 cases in group B, and 5 cases had PSQI > 5 points, and the prevalence rate was 50.00%. There were 53 cases in group C, 24 cases had PSQI > 5 points, and the prevalence rate was 45.3%. There were 10 cases in group D, 4 cases had PSQI > 5 points, and the prevalence rate was 40.00%. The statistical results are shown in Table 5.

For MHD patients with more serious underlying diseases, sleep quality is affected by more factors. HD alone cannot effectively improve various symptoms of patients, and there is no significant improvement in sleep quality. However, group A and group B are relatively effective in scavenging various medium and macromolecules and toxic substances. However, due to the high price and increased use of anticoagulants, not all patients can accept it. Therefore, clinically, an economical combination method can be selected, such as HD+HDF and HD+HDF+intermittent HP therapy. It can effectively solve the problem without significantly increasing the patient's economic burden and various side effects.

### 5.3. Effects of Dialysis Time Points on Sleep Quality

Due to the limitations of hemodialysis machines and venues, some maintenance dialysis patients need to arrange dialysis time until late. In order to determine whether different dialysis time points have an effect on sleep quality, this study divided 158 patients into a daytime group and a nighttime group. Among them, there were 104 patients on daytime dialysis, 65 patients had PSQI > 5 points, and the prevalence of sleep disturbance was 62.5%. There were 54 nocturnal dialysis patients, 32 patients had PSQI > 5 points, and the prevalence of sleep disorder was 59.26%. Compared between the two groups, it was found that there was no significant difference between the patients on daytime dialysis and those on nighttime dialysis (*P* > 0.05).

As shown in Figure 7, due to the lack of medical resources, the dialysis time of dialysis patients is limited by various factors such as venues and machines, and some dialysis patients need to perform nighttime dialysis. In order to compare the difference between day dialysis and night dialysis, this study compared day dialysis or night dialysis in maintenance hemodialysis patients and found no statistically significant difference between the two. Therefore, clinically, the dialysis time points of patients can be reasonably arranged according to the factors of each patient, such as distance and whether they need to work during the day.

### 5.4. Multivariate Analysis of Patients with Uremia

The sleep quality PSQI score of MHD patients was used as the dependent variable (PSQI > 5 was set as 1, PSQI ≤ 5 was set as 2), and the influencing factors of univariate analysis were used as independent variables. After assignment, multivariate logistic regression analysis was performed. The analysis results are shown in Tables 6 and 7.

With the aging of the domestic population and the increase of various diseases such as hypertension and diabetes, the number of CKD patients has increased year by year, and the resulting ESRD patients have also gradually increased. At the same time, due to the improvement of the social medical security system and the improvement of medical level, the survival time of uremia patients is prolonged. The quality of life of maintenance hemodialysis patients has become an important public health issue in the country. The incidence of CKD varies across regions, but both the prevalence and incidence are on the rise. The resulting prevalence of ESRD has also increased year by year. MHD patients have formed a huge group in society. The problem of sleep quality in MHD patients is affected by many factors, and many factors work together, resulting in poor sleep quality in MHD patients.

## 6. Conclusion

The sleep quality of MHD patients is affected by a variety of factors, and the incidence of sleep disorders is high. This paper further explores the factors that affect the quality of sleep in patients with uremia. The results of this study showed that the sleep quality of maintenance hemodialysis patients was affected by a combination of factors. The influencing factors listed in this article cannot explain all, and the probability of occurrence of each factor is different, and the severity of the impact is also different. Only from the influencing factors listed in this article, the study shows that during the dialysis period, the patient's weight gain, the selected dialysis method, the cholesterol level, the hemoglobin level, and the PTH level have the greatest impact on the sleep quality of MHD patients. It is an independent risk factor for sleep disturbance in patients with uremia.

## Figures and Tables

**Figure 1:** Schematic diagram of the principle of hemodialysis.

**Figure 2:** Schematic diagram of the patient's hemodialysis process.

**Figure 3:** Specific manifestations of sleep disorders.

**Figure 4:** The gender and age of patients and the composition of underlying diseases.

**Figure 5:** Changes in prevalence and *P* values.

**Figure 6:** Changes in *X*^2^/*P* of dialysis frequency and dialysis time in patients with uremia.

**Figure 7:** Effects of different dialysis time points on sleep quality.

**Table 1:** Effects of gender on sleep quality in patients with uremia.

Gender	Male	Female
Total	103	54
PSQI > 5 (%)	61.2 (62%)	32 (59.3%)
*X* ^2^	0	
*P* value	1	

**Table 2:** Effects of age on sleep quality in patients with uremia.

Age	Total	PSQI > 5 (%)
Group A (≤30)	14	6 (42.9%)
Group B (≥30, <45)	45	20 (44.4%)
Group C (>45, ≤60)	48	34 (70.8%)
Group D (>60, ≤75)	34	25 (73.5%)
Group E (>75)	17	12 (70.6%)

**Table 3:** Effect of monthly dialysis rate on sleep quality.

Monthly dialysis frequency	Total	PSQI > 5 (%)
Group A (2 times a week)	52	35 (67.3%)
Group B (5 times a fortnight)	33	16 (48.5%)
Group C (3 times a week)	75	45 (60%)

**Table 4:** Effect of dialysis time on sleep quality.

Monthly dialysis frequency	Total	PSQI > 5 (%)
Group A (>3 mon, ≤12 mon)	36	16 (44.4%)
Group B (>12 mon, ≤36 mon)	48	36 (75%)
Group C (>30 mon)	75	45 (60%)

**Table 5:** Effect of dialysis mode on sleep quality.

Dialysis method	Total	PSQI > 5 (%)	*X* ^2^	*P*
Group A	85	64 (75.3%)	*X* ^2^_AB_ = 5.6	*P*_AB_ = 0.018
Group B	10	5 (50%)	*X* ^2^_AC_ = 10.8	*P*_AC_ = 0.001
Group C	53	24 (45.3%)	*X* ^2^_AD_ = 9	*P*_AD_ = 0.003
Group D	10	4 (0%)	*X* ^2^_BC_ = 0.22	*P*_BC_ = 0.64
			*X* ^2^_BD_ = 0.22	*P*_BD_ = 0.64
			*X* ^2^_CD_ = 1.1	*P*_CD_ = 0.29
			*X* ^2^ = 17.3	*P* = 0.0006

**Table 6:** Grouping and assignment of each influencing factor.

Factor	Variable	Assign
Age	1	45 ~ 75 = 1, ≤45 and >75 = 2
Dialysis age	2	12 ~ 36 = 1, ≤12 and >36 = 2
Weight gain during dialysis	3	≥3 = 1, <3 = 1
Dialysis method	4	HD = 1
CHO	5	≥5.2 = 1, <5.2 = 2
HGB	6	≤70 = 1, >70 = 2
Calcium phosphorus product	7	≥55.8 = 1, <55.8 = 2
PTH	8	≤585 = 2, >585 = 1
BNP	9	≥400 = 1, <400 = 2
Are you diabetic	10	Yes = 1, no = 2
Is it RH	11	Yes = 1, no = 2
Sleep quality score (PSQL)	—	PSQI > 5 = 1, PSQI ≤ 5 = 2

**Table 7:** Prevalence score analysis table of uremia patients.

Influencing factors	*B*	Sig.	Exp(*B*)	95% CI	
				Lower limit	Upper limit
Age	0.76	0.12	2.15	0.81	5.65
Dialysis age	0.8	0.15	2.22	0.76	6.49
Weight gain during dialysis	1.98	0	7.62	2.74	19.28
Dialysis method	1.38	0.009	3.97	1.41	11.2
CHO	2.04	0.013	7.68	1.54	38.35
HGB	2.21	0.001	9.13	2.4	34.81
Calcium phosphorus product	-0.28	0.66	0.75	0.22	2.64
PTH	1.14	0.05	3.11	1.02	9.55
BNP	0.97	0.11	2.65	0.81	8.66
Are you diabetic	0.81	0.33	2.25	0.45	11.26
Is it RH	0.26	0.62	1.3	0.48	3.51

## Data Availability

No data were used to support this study.
